This article has been retracted.

# Nursing Observation on the Clinical Efficacy and Toxicity of Lobaplatin Compared with Cisplatin in the Treatment of Locally Advanced Hypopharyngeal Carcinoma Based on Intelligent CT Imaging

**DOI:** 10.1155/2021/9982888

**Published:** 2021-06-30

**Authors:** Yunyan Li, Guangrun Yang, Mengmeng Li, Xu Tong

**Affiliations:** Department of Radiotherapy, The Third Affiliated Hospital of Qiqihar Medical University, Qiqihar 161000, Heilongjiang, China

## Abstract

With the acceleration of people's life rhythm, the incidence of hypopharyngeal cancer has generally increased. This study mainly explores the clinical efficacy and toxicity of lobaplatin compared with cisplatin in the treatment of locally advanced hypopharyngeal carcinoma based on intelligent CT imaging. Group A received lobaplatin combined with docetaxel induction chemotherapy for 2 cycles after cisplatin combined with intensity-modulated radiotherapy. Lobaplatin was added to the patient, then, 200 ml of 5% glucose was added, and the patient was injected intravenously for 1.8 hours. After 2 cycles of induction chemotherapy, simultaneous lobaplatin chemotherapy was performed every week for 5 weeks (10 mg/week), and the efficacy was evaluated after 4 consecutive courses of treatment. Group *B* received cisplatin combined with docetaxel induction chemotherapy after 2 cycles of cisplatin combined with intensity-modulated radiotherapy. Group *C* was the control group and was not treated with cisplatin or docetaxel. Stomach protection treatment was given in time throughout the treatment process. All patients underwent normal CT (NCCT) and enhanced CT (CECT) examinations before treatment. We extracted 5 mm plain scan CTQNCCT and enhanced CT (CECT) digital DICOM images from the PACS system for omics feature selection. Toxic and side effects are rated in different degrees according to the evaluation criteria of the National Cancer Institute (NCD) common adverse events. Blood routine and liver and kidney function tests were checked every week, and the medication was stopped immediately if there is a serious reaction. In addition, in vitro cell culture was set up to test the inhibitory effect of cisplatin and lobaplatin on the proliferation of cancer cells. The incidence of digestive tract reaction was 13.0% in the A plan group and 58.3% in the B plan group. The A group was lower than the B group, and the difference was statistically significant (*P*=0.001 < 0.05). Compared with cisplatin, lobaplatin has a milder gastrointestinal reaction, and there is no common hepatic and renal toxicity of cisplatin. This study is helpful to provide guidance for the clinical efficacy of locally advanced hypopharyngeal cancer treatment.

## 1. Introduction

Squamous cell carcinoma is characterized by high aggressiveness, high early metastasis rate, high recurrence rate, and difficult early detection. Hypopharyngeal cancer is a relatively common tumor in otolaryngology head and neck surgery. Nowadays, the common treatment methods for hypopharyngeal cancer include surgery and subsequent radiotherapy and chemotherapy, but these common methods have more or less unavoidable side effects, such as the loss of throat function, and seriously affect the quality of life of patients after surgery. Despite the rapid development of surgical methods in recent years, the rate of distant metastasis and recurrence has not changed significantly.

Radiotherapy and chemotherapy can reduce the distant metastasis rate of cancer cells and can transform it into survival benefits. Through subgroup analysis, the benefits of chemotherapy mainly come from concurrent chemotherapy. There are many options for concurrent chemotherapy for hypopharyngeal cancer, such as platinum single-agent, paclitaxel single-agent, tigeo single-agent, platinum-based combined with fluorouracil, platinum-based combined with paclitaxel, and other combined drugs. Platinum antitumor drugs can act on the entire cell cycle and inhibit the proliferation of cancer cells. Compared with combination chemotherapy, platinum-based single-drug regimens have lower toxicity and better tolerability.

An optimized attenuation compensation and contrast enhancement algorithm can improve the quality of intravascular optical coherence tomography (IVOCT) images and overcome the shortcomings of previous algorithms, including artifacts such as tissue attenuation and changes in artifact shadows. Zhou first theoretically analyzed the changes in tissue attenuation caused by compensation and enhancement. He compared the estimated tissue attenuation values in the baseline and enhanced IVOCT images with calcium, lipid, or fibrous plaques to find the best enhancement coefficient that retains the attenuation characteristics. Then, he compared IVOCT images with different enhancement coefficient values to evaluate the effect of each algorithm based on the improvement of depth visibility, contrast enhancement, and feature retention. Although his research can derive the best attenuation coefficient for attenuation compensation and contrast enhancement algorithms, the research lacks systematic contrast [1]. KouvAa aims to compare the diagnostic accuracy of axial chest CT, other imaging techniques, and image reconstruction algorithms with fiberoptic bronchoscopy (FOB) endoscopy in patients with newly discovered endobronchial lesions. He conducts retrospective and prospective research on the literature. The articles considered included patients with intrabronchial stenosis; regardless of whether they received image reconstruction techniques, all underwent chest-thoracic computed tomography and fiberoptic bronchoscopy. 10 PubMed or CancerLit published 10 studies (6 prospective/4 retrospective studies) which were included in the research criteria. A total of 633 patients participated in the study, and another 53 patients were included in the control. All patients underwent fiberoptic bronchoscopy (FOB) and chest imaging. Although his research has the same sensitivity as fiberoptic bronchoscopy for most imaging techniques, it has a significant negative predictive value [2]. Benjamin aims to determine whether the use of analytical morphology (AM) for comprehensive image analysis in risk-stratified pancreatic surgery patients is to enhance or replace the geriatric assessment (GA). One hundred and thirty-four pancreatic surgery patients were identified from the prospective cohort. The 63 patients in this cohort underwent preoperative CT scans in addition to a comprehensive geriatric evaluation. AM was used to process CT scans. Univariate analysis and a robust elastic net model were used to evaluate the relationship with the severe complications of the National Surgical Quality Improvement Program (NSQIP). Although his research can conclude the relationship between severe complications of NSQIP and low psoas major, low-density (0 to 30 HU) psoas major area, visceral fat HU, visceral fat area, and subcutaneous fat HU, the research process is too complicated [3]. Luckenbaugh evaluated the relationship between psoas muscle area and short-term recovery after radical cystectomy. After identifying the patients undergoing radical cystectomy, he used the established analytical morphology technique to stage the computed tomography to calculate the area of the psoas major muscle. Then, using a validated CARE questionnaire (27 items divided into four areas (activity, cognition, gastrointestinal, and pain recovery)), he determined the psoas major and low psoas muscle areas The patient is early recovered. Finally, he used a nested linear regression model to evaluate the relationship between psoas muscle area and changes in CARE score. Although his research may be an important predictor of preoperative recovery for women undergoing radical cystectomy, it has never been in a broader sense; analyzing morphology may be a novel method to better understand perioperative risks [4].

This study mainly explores the clinical efficacy and toxicity of lobaplatin compared with cisplatin in the treatment of locally advanced hypopharyngeal carcinoma based on intelligent CT imaging. Group A received lobaplatin combined with docetaxel induction chemotherapy for 2 cycles after cisplatin combined with intensity-modulated radiotherapy. Group B received cisplatin combined with docetaxel induction chemotherapy after 2 cycles of cisplatin combined with intensity-modulated radiotherapy. Group *C* was the control group and was not treated with cisplatin or docetaxel. Stomach protection treatment was given in time throughout the treatment process. All patients underwent normal CT (NCCT) and enhanced CT (CECT) examinations before treatment. We extracted 5 mm plain scan CTQNCCT and enhanced CT (CECT) digital DICOM images from the PACS system for omics feature selection. Toxic and side effects are graded in different degrees according to the evaluation criteria of common adverse events. Blood routine and liver and kidney function tests were checked every week, and the medication was stopped immediately if there is a serious reaction. In addition, in vitro cell culture was set up to test the inhibitory effect of cisplatin and lobaplatin on the proliferation of cancer cells.

## 2. Clinical Efficacy of Hypopharyngeal Cancer Treatment

### 2.1. Intelligent CT Imaging Omics

The quantitative image features used in radiomics are based on the density, shape, size, and texture determined by the phenotype and microenvironment information of the lesion so that the image can be quantitatively analyzed to reflect the complexity and variation of the lesion [5, 6]. The morphology of low-risk lesions is mostly regular, round, or quasicircular, while the morphology of high-risk lesions is mostly lobed or irregular. The corresponding model establishment is required for CT technology detection, and image processing is particularly important at this time [7]. The formula for the color change with the corner when shooting is

(1) $$\begin{array}{c} f=mc^{h}\sin\theta . \end{array}$$

In the formula, the shooting color change *f* starts to change with the turning angle as an odd function. Due to the limitation of the shooting space, the shooting image always fluctuates within a certain range [8, 9]. Pay attention to the reflective characteristics of the image when shooting.

(2) $$\begin{array}{c} F=e\left(m^{h}c^{h}+m^{j}c^{k}\right). \end{array}$$

It can be seen from the above formula that the reflective characteristics of *F* are superimposed on each other, so pay attention to the changes on the front and back when shooting [10]. The first-order conversion of reflective characteristics is as follows:

(3) $$\begin{array}{c} S_{x}=\left(em^{b}c_{x}+emb_{x}\right)\left|c^{d}\right|. \end{array}$$

The above formula reflects the change of edge corner area *S*_*x*_ in the calculation of reflective characteristics [11]. The window period change *S*_c_ is [12]

(4) $$\begin{array}{c} S_{c}=p\left(em^{b}c_{x}-emb_{x}\right)\left|c^{d}\right|+c^{k}. \end{array}$$

The direction change *O*_*x*_ of the specular reflection is [8]

(5) $$\begin{array}{c} O_{x}=\left(f_{x}+c_{h}\right)f. \end{array}$$

Reflective intensity *E*_*c*_is

(6) $$\begin{array}{c} E_{c}=\left(\frac{p\left(em^{b}c_{x}-emb_{x}\right)\left|c^{d}\right|}{b}\right)+c^{k}*m. \end{array}$$

The ratio of saturation to the light source *λ*_*c*_is

(7) $$\begin{array}{c} \lambda_{c}=\frac{p\left(em^{b}c_{x}-emb_{x}\right)b}{ev^{b}c_{x}0-evb_{x}}. \end{array}$$

### 2.2. Cisplatin and Lobaplatin

Lobaplatin is equivalent to or better than the first-generation DDP and the second-generation CBP, has no cross-resistance to cisplatin (DDP), and has similar side effects to carboplatin (CBP). Due to the poor tolerance of cisplatin chemotherapy, drug resistance or short-term recurrence occurs after chemotherapy, and the long-term survival rate is low. Therefore, exploring new combined chemotherapy regimens has become a research hotspot in recent years. The main adverse drug reaction of lobaplatin is thrombocytopenia [13]. At present, there is no standard chemotherapy regimen for neoadjuvant chemotherapy for cervical cancer. Current reports are more common in BVP, TIP, PT, etc. Currently, platinum-based chemotherapy regimens are still one of the treatment options for patients with local IB2-IIB stage cervical cancer. There are many commonly used antitumor chemotherapy drugs; cisplatin (DDP) is one of them, especially in the treatment of head and neck tumors [14, 15]. However, due to the weak selectivity of chemotherapeutic drugs for acting cells, it is unavoidable that while chemotherapeutic drugs act on tumor drugs, they will also cause different degrees of damage to the normal tissue cells of the human body. In addition, because of their application more extensively, tumor cells began to develop resistance to cisplatin, which greatly restricted the general application of the cisplatin. Therefore, finding an efficient method to reduce the resistance of cisplatin and increase the sensitivity of patients to chemotherapy drugs to improve the efficiency of chemotherapy is the main direction of current research [16]. Looking at the foregoing, we can find that there are many unavoidable problems in the current conventional treatment methods for tumors. Whether from the treatment effect or the impact after treatment, it can be found that these treatment methods have a huge impact on patients. For tumors, the application of gene therapy combined with chemotherapeutic drugs is a new treatment direction that has been proposed in recent years. This gene-combined chemotherapy treatment method neither damages the integrity of human tissues like surgery nor causes unbearable damage to normal human tissues like radiotherapy, and it does not even cause patients to apply chemotherapy drugs like chemotherapy. After that, there is still no obvious antitumor effect. On the contrary, the comprehensive treatment method of gene combined chemotherapy is only to transfer the suicide gene or tumor suppressor gene into the local tumor cells, so that it can be stably expressed in the tumor cells, so it can play a highly effective antitumor effect to achieve the cure of the tumor (purpose [17, 18]). The molecular formulas of lobaplatin and cisplatin are shown in Figure 1.

### 2.3. Hypopharyngeal Cancer

At present, surgical resection is still one of the main methods for the treatment of hypopharyngeal cancer. The main objectives of surgical treatment are as follows: complete removal of the tumor and providing a proper safety margin, proper preservation of laryngeal function, reconstruction of the pharyngeal cavity and upper gastrointestinal tract, and removal of cervical lymph node metastases. The role of radiotherapy has the following aspects: eliminate smaller and sensitive hypopharyngeal tumors; provide a wider range of safety beyond the surgical margin; control subclinical lesions in the neck to avoid neck dissection; for difficult surgical resection, the lesions may be removed after radiation; palliative radiotherapy is used for patients who refuse to operate or cannot be operated on. Regarding the combination of radiotherapy and surgery, in terms of the timing of radiotherapy, most of them are currently postoperative radiotherapy; however, there is no significant difference in survival rate between preoperative or postoperative radiotherapy [19, 20].

In the CT detection process of cancer, suppose that the gray value of the image *f* is *I*; then, the total pixels are [21]

(8) $$\begin{array}{c} X=\sum_{i=1}^{L}\left(x_{1}+x_{2}+\cdots +x_{n}\right). \end{array}$$

The probability of each gray level *p* is

(9) $$\begin{array}{c} p=\left(\frac{n_{1}}{N}*\frac{1}{B}\right)\sum_{i=1}^{m}m^{2}. \end{array}$$

Suppose that the image is divided into two regions with gray *k* as the threshold; then [22]

(10) $$\begin{array}{c} \omega_{A}=\sum_{i=1}^{k}p_{i},\\ \omega_{B}=\sum_{i=k+1}^{L}p_{i}. \end{array}$$

The average gray level of regions A and B is [23]

(11) $$\begin{array}{c} Q_{A}=\frac{1}{\omega }\sum_{i=1}^{k}\text{m}*p_{i}+\left(\frac{Q\left(k\right)}{\omega \left(k\right)}\right),\\ Q_{B}=\frac{1}{\omega }\sum_{i=k+1}^{L}i*p_{i}=\left(\frac{Q-Q\left(k\right)}{1-\omega \left(k\right)}\right). \end{array}$$

Among them, *Q* is the average gray level of the whole image [24, 25].

(12) $$\begin{array}{c} Q=\sum_{i=1}^{L}i*p_{i}=\left(\omega_{A}Q_{A}+\omega_{B}Q_{B}\right). \end{array}$$

For tumor gene therapy, it refers to the application of certain gene transfer technologies, such as retrovirus-mediated gene technology, to introduce target genes that can perform specific functions into target cells [26]. Therefore, in addition to the current conventional treatments, a better understanding of the process of tumor occurrence and development can increase the possibility that gene therapy will become another new treatment method for hypopharyngeal cancer. Moreover, hypopharyngeal cancer shows low sensitivity to anticancer drugs, and its underlying mechanism is still unknown, which also leads to a poor prognosis and a low five-year survival rate for patients with hypopharyngeal cancer [27, 28]. Therefore, research and development of new treatment methods to reduce the antichemotherapy effect of hypopharyngeal cancer and improve its five-year survival rate are considered to be a new challenge [29]. The variance *σ*^2^ of the two regions is

(13) $$\begin{array}{c} \sigma^{2}=Q_{A}{\left(\theta_{A}-\theta \right)}^{2}+Q_{B}{\left(\theta_{B}-\theta \right)}^{2}=\left(\frac{\mu Q\left(k\right)-\lambda \left(k\right)}{Q\left(k\right)\left(1-Q\left(k\right)\right)}\right). \end{array}$$

Change K from 1 to *L* according to the criterion of maximum variance between classes [30].

## 3. Lobaplatin versus Cisplatin in the Treatment of Locally Advanced Hypopharyngeal Carcinoma

### 3.1. Research Objects and Standards

#### 3.1.1. Patient Information

There are 59 patients. The male to female ratio is 1 : 1. The age ranges from 38 to 72 years old, with the average age being 57.9; pathology is locally advanced hypopharyngeal carcinoma; all patients were treated for the first time; liver and kidney functions were normal before medication; all patients had the following examinations before treatment: electronic rhinopharyngeal endoscopy. All patients signed an informed consent form.

#### 3.1.2. Inclusion Criteria

With reference to the ICD-10 disease diagnosis code, the medical record retrieval system of our hospital and the paper-based medical records were used to retrieve the data of hypopharyngeal cancer patients admitted to this hospital from February 2019 to January 2020. Based on the third edition of the International Classification of Tumors based on the diagnostic criteria for multiple primary cancers established in the Handbook and combined with actual clinical conditions, the following inclusion and exclusion criteria are formulated:

1. Hypopharyngeal cancer and esophageal cancer are confirmed by histopathology as squamous cell carcinoma
2. Each cancer foci have its own pathological morphology
3. Each patient's hypopharyngeal cancer and esophageal cancer can occur simultaneously or sequentially, but there is no affiliation between two or more tumors and cancer must be separated from normal tissues, that is, it is not directly spread by one to form another
4. The clinical data is relatively complete, and data analysis and follow-up are available

#### 3.1.3. Exclusion Criteria

1. The tumors are continuous with each other or the possible cases of metastasis cannot be excluded.
2. The clinical diagnosis time is too short (<1 month).
3. The clinical data is severely lacking, and data analysis and follow-up cannot be carried out. The TNM staging of hypopharyngeal carcinoma is shown in Table 1.

### 3.2. Treatment Plan

#### 3.2.1. Group A

Lobaplatin was combined with docetaxel induction chemotherapy 2 cycles after cisplatin combined with intensity-modulated radiotherapy. On the first day, the patient was given docetaxel 70 mg/m^2^, mixed with 200 ml of normal saline, and injected into the vein for 1.8 hours; on the second day, lobaplatin (35 mg/m^2^) was added, and then, 5% glucose (200 ml) was added and injected into the vein for 1.8 hours continuously. The duration of one treatment cycle was set to 15 days. After 2 cycles of induction chemotherapy, simultaneous lobaplatin chemotherapy was performed every week for 5 weeks (10 mg/week), and the efficacy was evaluated after 4 consecutive courses of treatment.

#### 3.2.2. Group B

Induction chemotherapy with cisplatin combined with docetaxel was performed after 2 cycles of cisplatin combined with intensity-modulated radiotherapy. On the first day, the chemotherapy drugs were mixed with 200 ml of normal saline and injected intravenously for 1 hour; on days 2-3, 30 mg/m^2^ of cisplatin was added, mixed with 200 ml of normal saline, and injected intravenously for continuous infusion for 1.8 hours. The time of 1 treatment cycle was set as 15 days; after 2 cycles of induction chemotherapy, simultaneous chemotherapy was done with a cisplatin weekly regimen for 5 weeks (10 mg/week), and the curative effect was evaluated after 4 consecutive courses of treatment.

#### 3.2.3. Group C

This group is the control group, without cisplatin or docetaxel treatment. Two cycles of docetaxel induction chemotherapy were followed by radiotherapy. On the first day, the chemotherapy drugs were mixed with 200 ml of normal saline and injected into the vein for continuous infusion for 1 hour; on days 2-3, 200 ml of normal saline was added and injected into the vein for 1.8 hours for continuous infusion, setting 1 treatment. The cycle time is 15 days. After 2 cycles of induction chemotherapy, the therapeutic effect is evaluated after 4 consecutive courses of treatment.

Stomach protection treatment was given in time throughout the treatment process. Until the disease progresses, intolerable toxicity appears, or the patient requests the termination of chemotherapy, up to 6 cycles of chemotherapy.

### 3.3. CT Image Acquisition

All patients underwent normal CT (NCCT) and enhanced CT (CECT) examinations before treatment. We extracted 5 mm plain scan CTQNCCT and enhanced CT (CECT) digital DICOM images from the PACS system for omics feature selection. Multiplanar reconstruction (MPR) is used to determine the edge of the tumor in 1.25 mm and 2.5 mm thick images. The enhanced CT scan used in this study is a 64-channel or more than 8-channel detector CT scanner (LightspeedUItra GE Healthcare). In the conventional neck scan CT (NCCT), 70 ml of iodine contrast agent (Ultravist370 BayerScheringPharma) was injected intravenously (flow rate 3.0 ml/s) with a high-pressure syringe for enhanced CT scan. After the injection of the contrast agent, after a delay of 25 seconds and 60 seconds, all enhanced CT (CECT) images were obtained. In this study, only an enhanced CT scan with a delay of 60 seconds (venous phase) was selected for image analysis. The scanning parameters are as follows: 120 kV, 260 mA, rotation time of 0.6 s or 0.8 s, probe collimator of 64 *∗* 0.625 mm or 8 × 0.625 mm, field of view (FOV) of 320 × 320 mm, and matrix of 512 × 512.

### 3.4. Toxic and Side Effects

Toxic and side effects can be evaluated after completing a cycle of chemotherapy. Toxic and side effects are rated in different degrees according to the evaluation criteria of the National Cancer Institute (NCD) common adverse events. Blood routine and liver and kidney function tests were checked every week, and the medication was stopped immediately if there is a serious reaction. Then, the follow-up time is 10 months, and the prognosis consultation is carried out by telephone and e-mail.

### 3.5. Cell Culture In Vitro

FaDu cells in the logarithmic growth phase (density: 1 × 10%/mL) were seeded on 96-well culture plates. It was observed that all the cells were attached to the glass wall. The experiment is divided into three groups: zero control group (100 *μ*1 medium without cells), contrast group (normal cell culture containing (0.2, 0.4, 0.6, and 0.8 *μ*g/mL) lobaplatin), and experimental group (0.2, 0.4, 0.6, and 0.8 *μ*g/mL cisplatin); each group has 3 complex culture holes. The cell culture plate was put into the original cell incubator and incubate for another 48 hours. After removing the agent, 20 *μ*l of MTT solution was added to each incubate in the well for 4 hours. 150 *μ*L of DMSO solution was added to each well and mixed thoroughly after shaking. A microplate analyzer was used to calculate the absorbance of the cells and the degree of inhibition of growth.

### 3.6. Statistical

According to RECIST1 to assess the degree of remission of the tumor after treatment, we have the following: complete CR (complete disappearance of all target lesions), partially effective PR (at least 30% reduction in target lesions), and stable SD (PR and PD) and PD (target lesions or new; the lesion has increased by at least 20%). Harmful reactions are classified according to NCI-CTCAE4.0. The statistical software SPSS23.0 and the Kaplan–Meier method were used in the analysis. Regarding the tumor remission rate, the maintenance rate of laryngeal function, and the incidence of adverse reactions and descriptive statistics were used. The impact of prognosis on overall survival was investigated. The classification count data uses the chi-square test, the measurement data uses the *t*-test, and the rank data uses the order and test. When the test level *α* = 0.05 and *P* < 0.05, the difference is considered statistically significant.

## 4. Results and Discussion

### 4.1. Toxic Side Effects

59 patients were randomly selected from the AB groups for statistics. Both groups A and B can be evaluated for adverse reactions, and there is no chemotherapy-related death. The main toxic and side effects were bone marrow suppression and gastrointestinal reactions. The gastrointestinal reactions were mainly nausea and vomiting, and most of them could be relieved after symptomatic treatment, reduced dose chemotherapy, or delayed chemotherapy. There was 1 case in group A (4.3%), program B. One patient (2.8%) in the group was unable to tolerate severe side effects and stopped chemotherapy. There was no statistically significant difference between the two groups (*P*=0.745 > 0.05). Other side effects, such as liver damage and hair loss, are all mildly tolerable, and symptomatic treatment can be alleviated, and there was no effect on chemotherapy.

Myelosuppression: the incidence of leukopenia was 69.6% in group A and 91.7% in group B. Group A was lower than group B, and the difference was statistically significant (*P*=0.027 < 0.05). The incidence of anemia was 43.5% in the A plan group and 27.8% in the B plan group. The A group was higher than the B group, and the difference was not statistically significant (*P*=0.214 > 0.05). The incidence of thrombocytopenia was 43.5% in the A plan group and 19.4% in the B plan group. The A group was higher than the B group, and the difference was statistically significant (*P*=0.047 < 0.05).

The incidence of digestive tract reaction was 13.0% in the A plan group and 58.3% in the B plan group. The A group was lower than the B group, and the difference was statistically significant (*P*=0.001 < 0.05). The incidence of liver damage was 26.1% in the A plan group and 25.0% in the B plan group. The A group was higher than the B group, and the difference was not statistically significant (*P*=0.925 > 0.05). The incidence of hematuria (including microscopic hematuria and gross hematuria) was 4.3% in group A and 5.6% in group B. Group A was lower than group B, and the difference was not statistically significant (*P*=0.837 > 0.05). The incidence of proteinuria was 8.7% in group A and 5.6% in group B. Group A was higher than group B, and the difference was not statistically significant (*P*=0.640 > 0.05). The incidence of hair loss was 8.7% in plan A and 8.3% in plan B. Group A was higher than group B, and the difference was not statistically significant (*P*=0.961 > 0.05). There was no increase in creatinine, ototoxicity, or peripheral neurotoxicity. Compared with cisplatin, the gastrointestinal reaction of lobaplatin is lighter, and it has no liver and kidney toxicity, neurotoxicity, and ototoxicity common to cisplatin and does not require hydration. It has better adaptability in some tumors. The statistics of side effects are shown in Table 2. The statistical analysis of side effects is shown in Figure 2. The tumor suppressor mechanism of cisplatin is shown in Figure 3.

Platinum anticancer drugs have an effect on the entire cell cycle and may hinder the proliferation and cell viability of tumor cells. They have a wide range of anticancer and high activity and can play a very good role in combination with chemotherapy. Platinum anticancer agents are now considered to be relatively excellent chemotherapy and radiotherapy drugs. Cisplatin, due to its unique radiotherapy effect, is mainly cancer cells that play a synergistic effect due to the repair of damaged cells or obstruction of synchronization. At present, cisplatin is the most effective treatment for local hypopharyngeal cancer, but cisplatin has a relatively large gastrointestinal reaction and nephrotoxicity, which will affect the patient's tolerance. As the third-generation platinum drug docetaxel, the main dose-limiting toxicity is thrombocytopenia. Most clinical trials have shown that a single dose of docetaxel has immune activity against esophageal cancer, hypopharyngeal cancer, and other tumors. For the incidence of leukopenia, grades 1, 2, 3, and 4 were 4.3%, 26.1%, 26.1%, and 13.0% in group A and 2.8%, 13.9%, 36.1%, and 38.9% in group B. In the comparison between the two groups, the grade 4 group A was lower than the group B, and the difference was statistically significant (*P*=0.033 < 0.05); the difference in grades 1, 2, and 3 was not statistically significant (*P* > 0.05). For the incidence of leukopenia, grades 1-2 and 3-4 were 30.4% and 39.1% in group A and 16.7% and 75.0% in group B. In the comparison between the two groups, the 3-4 grade A group was lower than the B group; the difference was statistically significant (*P*=0.006 < 0.05); the 1-2 grade difference was not statistically significant (*P* > 0.05). The statistics of the incidence of leukopenia are shown in Table 3. The CT performed by the patient during the side effects is shown in Figure 4.

The pathology of patients with hypopharyngeal cancer is shown in Figure 5. When the patient swallows rough or overheated, irritating food, there will be intermittent pain. The pain is manifested as burning, acupuncture, and stretching, which can be temporarily relieved with antispasmodics.

The effect of cisplatin and lobaplatin on hypopharyngeal cancer cells can inhibit the proliferation of the cells. Multifactor analysis of variance showed that the concentration factor has an effect on the cell survival rate (*F* = 132.998, *P* < 0.001); the duration of action has an effect on the cell survival rate. There is an effect (*F* = 251.265, *P* < 0.001). After the same dose of cisplatin and lobaplatin act on hypopharyngeal cancer cells, the cell lethality rate in the cisplatin culture dish is 5%, and the lethality rate of lobaplatin is only 1.22%. The comparison shows that lobaplatin is less toxic to cells. The inhibitory effect of cisplatin is time-concentration-dependent, and the IC50 concentration of cisplatin alone for 48 h is 3.996 ug/ml. The hypopharyngeal carcinoma cells under the electron microscope are shown in Figure 6. The inhibition of cisplatin and lobaplatin on the growth rate of hypopharyngeal cancer cells is shown in Figure 7.

The expressions of apoptosis-related proteins Bax, Bcl-2, caspase-3, cleaved-caspase-3, and PI3K/AKT signaling pathway proteins were analyzed. The experiment was divided into a control group and a lobaplatin administration group. From the experimental results, it can be seen that the expression of Bax in T24 cells in the lobaplatin administration group increased, the expression of Bcl-2 decreased, cleaved-caspase-3/caspase-3 increased, PI3K in the PI3K/AKT signaling pathway decreased, and the P-Akt/Akt decreased; the related protein expression in ScaBER cells changed in the same trend. The results showed that lobaplatin promotes cell apoptosis by promoting the expression of apoptotic proteins and inhibits the expression of the PI3K/AKT signaling pathway to promote cell apoptosis. RT-PCR detection of apoptosis gene expression in the FaDu cell line is shown in Figure 8.

### 4.2. Imageomics Evaluation and Analysis

This survey will use ITK-SAP software (open source software, version 2.2.0). The area of interest (ROI) is drawn along the boundaries of each layer of the pharyngeal carcinoma block on the NCCT and CECT DICOM images. Next, after segmenting the region of interest (VOI), the features of the quantitative image are extracted. The tumor area was manually intercepted by a radiologist with 10 years of experience and then confirmed by the deputy chief radiologist of the hospital with 15 years of experience in head diagnosis. Moreover, for the segmentation and refinement of tumors, it is necessary to avoid images of residual cartilage (cracking cartilage, etc.). The CT image of arytenoid cartilage is shown in Figure 9.

As of the follow-up time, 50 patients were selected for investigation. The patients received a total of 20 chemotherapies, with an average of about 3 times per case. A total of 31 patients in group A underwent 74 operations, 29 patients (93.5%) received cisplatin and the bleeding was initially controlled, and 18 patients (58.1%) did not reappear hypopharyngeal dysfunction during the follow-up period; 19 patients in group B received lobaplatin after treatment, the bleeding was successful in the early stage (100%), 9 patients (47.4%) were successful in the late stage, and there was no significant difference in the control rate of the throat between the two groups (*P*=0.271, 0.461). Compared with cisplatin, lobaplatin has lower renal, neurological, or ototoxic side effects, and lobaplatin can overcome the cisplatin resistance produced by cancer cells. The CT image comparison of lobaplatin and cisplatin treatment is shown in Figure 10.

## 5. Conclusion

This study mainly explores the nursing observation of the clinical efficacy and toxicity of lobaplatin compared with cisplatin in the treatment of locally advanced hypopharyngeal carcinoma based on intelligent CT imaging. Group A received lobaplatin combined with docetaxel induction chemotherapy for 2 cycles after cisplatin combined with intensity-modulated radiotherapy. Group B received cisplatin combined with docetaxel induction chemotherapy after 2 cycles of cisplatin combined with intensity-modulated radiotherapy. Group *C* was the control group and was not treated with cisplatin or docetaxel. Stomach protection treatment was given in time throughout the treatment process. All patients underwent normal CT (NCCT) and enhanced CT (CECT) examinations before treatment. We extracted 5 mm plain scan CTQNCCT and enhanced CT (CECT) digital DICOM images from the PACS system for omics feature selection. Toxic and side effects are rated in different degrees according to the evaluation criteria of the National Cancer Institute (NCD) common adverse events. Blood routine and liver and kidney function tests were checked every week. The medication was stopped as soon as there is a serious reaction. In addition, in vitro cell culture was set up to test the inhibitory effect of cisplatin and lobaplatin on the proliferation of cancer cells. The incidence of digestive tract reaction was 13.0% in the A plan group and 58.3% in the B plan group. The A group was lower than the B group, and the difference was statistically significant (*P*=0.001 < 0.05). Compared with cisplatin, lobaplatin has a milder gastrointestinal reaction, and there is no common hepatic and renal toxicity of cisplatin. This study is helpful to provide guidance for the clinical efficacy of locally advanced hypopharyngeal cancer treatment.

## Figures and Tables

**Figure 1:** Molecular formula of lobaplatin and cisplatin (lobaplatin http://alturl.com/z5bk7, cisplatin http://alturl.com/i64f7). (a) Lobaplatin. (b) Cisplatin.

**Figure 2:** Statistical analysis of side effects.

**Figure 3:** Cisplatin anticancer mechanism (http://alturl.com/occy3).

**Figure 4:** CT performed by the patient during toxic side effects (http://alturl.com/w6p6w).

**Figure 5:** Pathology of patients with hypopharyngeal cancer (http://alturl.com/p6dmc).

**Figure 6:** Hypopharyngeal cancer cells under electron microscope (http://alturl.com/s5xmt).

**Figure 7:** Cisplatin and lobaplatin inhibit the growth rate of hypopharyngeal cancer cells.

**Figure 8:** RT-PCR detection of apoptotic gene expression in FaDu cell line (http://alturl.com/phrqp).

**Figure 9:** CT image of arytenoid cartilage (http://alturl.com/kcfxm).

**Figure 10:** Comparison of CT images of lobaplatin and cisplatin treatment (http://alturl.com/gjyo6). (a) Lobaplatin treatment. (b) Cisplatin treatment.

**Table 1:** TNM staging of hypopharyngeal carcinoma.

Primary tumor (*T*)	Symptom description
Tx	Primary tumor cannot be assessed
T0	No evidence of primary tumor
Tis	Carcinoma in situ
T1	An anatomical subregion of the pharynx with a maximum diameter of 2 cm

**Table 2:** Statistics of side effects.

Toxic side effects	A	B	*P*
Leukopenia	16 (69.6)	33 (91.7)	0.027
Anemia	10 (43.5)	10 (27.8)	0.214
Thrombocytopenia	10 (43.5)	7 (19.4)	0.047
feA sick and vomit	3 (13.0)	21 (58.3)	0.001
Increased liver function ALT/AST	6 (26.1)	9 (25.0)	0.925
Increased creatinine	0 (0)	0 (0)	<0.001
Hematuria	1 (4.3)	2 (5.6)	0.837
Proteinuria	2 (8.7)	2 (5.6)	0.640
Hair loss	2 (8.7)	3 (8.3)	0.961

**Table 3:** Leukopenia incidence statistics.

Groups	*n*	1	2	3	4	1-2	3-4
A	23	1 (4.3)	6 (26. 1)	6 (26.1)	3 (13.0)	7 (30.4)	9 (39.1)

B	—	1 (2.8)	5 (13.9)	13 (36.1)	14 (38.9)	6 (16.7)	27 (75.0)

## Data Availability

No data were used to support this study.
